# Applying Internet information technology combined with deep learning to tourism collaborative recommendation system

This article has been retracted.

**DOI:** 10.1371/journal.pone.0240656

**Published:** 2020-12-03

**Authors:** Meng Wang

**Affiliations:** School of Economics and Trade, Henan University of Engineering, Henan, Zhengzhou, China; University College London, UNITED KINGDOM

## Abstract

Recently, more personalized travel methods have emerged in the tourism industry, such as individual travel and self-guided travel. The service models of traditional tourism limit the diversity of service options and cannot fully meet the individual needs of tourists anymore. The aim is to integrate sparse tourism information on the Internet, thereby providing more convenient, faster, and more personalized tourism services. Based on the shortcomings of the traditional tourism recommendation system, a deep learning-based classification processing method of tourism product information is proposed. This method uses word embedding in the data preprocessing stage. The Convolutional Neural Network (CNN) is used to process review information of users and tourism service items. The Deep Neural Network (DNN) is used to process the necessary information of users and tourism service items. Also, factorization machine technology is used to learn the interaction between the extracted features to improve the prediction model. The results show that the proposed model can maintain an excellent precision of 64.2% when generating personalized recommendation lists for users. The sensitivity and accuracy of the recommendation list are better than other algorithms. By adding DNN, the word embedding method, and the factorization machine model, the precision is improved by 30%, 33.3%, and 40%, respectively. The model accuracy is the highest with 40 hidden factors, 100 convolutions, and a 100+50 combination hidden layer. Compared with traditional methods, the proposed algorithm can provide users with personalized travel products more accurately in personalized travel recommendations. The results have enriched and developed the theory of tourism service supply chain, providing a reference for constructing a personalized tourism service system.

## 1. Introduction

As the economy grows, people’s living standards have been improved, and tourism has gradually become one of the fastest-growing industries all around the world [1]. Tourism is centered on travel agencies, which have occupied the mainstream of the tourism consumer market for a long time. However, many shortcomings have also been exposed during these long-term operations [2]. With the rapid development of the mobile Internet, cloud computing, big data, and artificial intelligence, the tourism industry and the computer industry are becoming more closely integrated [3]. People can search for all kinds of tourism service information more conveniently and quickly, while enjoying the convenience brought by information technology [4]. However, with the advent of the big data era, information relating to tourism products has grown exponentially, and information resources are becoming more diverse [5]. Due to the massive amount of information, resulting in information overload, people are unable to choose quickly and accurately [6]. Especially with the rapid growth of the tourism industry, major Internet companies have joined in one after another, which is troublesome for tourists, and leads to extremely low efficiency [7]. In addition, the wide distribution of Internet resources makes it difficult for users to find the information they need [8]. Due to the lack of theoretical and technical support, Internet travel service providers cannot currently provide customized service products based on the individualized needs of tourists [9]. Therefore, to cope with this information overload phenomenon and solve problems in the tourism recommendation service, it is essential to use Internet information technology and other new ways to implement personalized recommendations.

As an excellent algorithm for classifying and processing data, deep learning overcomes traditional singular and mechanical data processing methods. It can learn and analyze the data thoroughly [10]. In recent years, many scholars worldwide have applied deep learning technology to the tourism industry. Yin et al. (2017) used deep learning technology to propose a spatially-aware hierarchical collaborative deep learning model; this model employed deep learning of personalized information from the perspective of heterogeneous features to layer spatially-aware personal preferences, which effectively eliminated the problem of data sparseness in travel service recommendation [11]. Guo et al. (2018) analyzed the user’s travel behavior in detail and developed a deep learning model to integrate geographic and social influences for personalized travel recommendation services, using a semi-restrictive Boltzmann machine to model the geographic similarity and the conditional layer to model the social impact; the experimental results showed that this method had better performance than other latest methods [12]. Chen et al. (2020) adopted an unsupervised deep learning model to embed personalized recommendation text content and then proposed a personalized travel recommendation model that seamlessly integrated the embedded text content with traditional and widely-used user access categories for effective prediction of user interest [13]. Lee et al. (2020) proposed a travel route recommendation system based on a Gated Recurrent Unit (GRU) network and RNN algorithm, which improved the performance of personalized travel recommendation by integrating Bayesian personalized ranking error functions [14]. The above results suggest that the combination of computers and the tourism industry is often used to predict the number of tourists, and more models are being established to facilitate the local tourism service department to prepare for the response. However, there have been few investigations into personalized recommendations of tourism products.

Therefore, it is necessary to solve the problems in the tourism recommendation system and improve the ability to make personalized recommendations of travel products. Through deep learning technology and the review information available for travel products on major tourism platforms, word embedding is combined with factorization machine technology to propose a new method of classification processing of tourism product information. This method can deeply mine the information features of user reviews on all network platforms to find a deeper meaning. This investigation can effectively classify and process online tourism product data to meet the need for personalized recommendations of tourism services.

## 2. Methods

### 2.1 Travel recommendation and Internet information technology

(1) Travel recommendation system: currently, Internet companies making presentations for the tourism industry provide users with various tourism products. At the same time, users generate a series of data every day [15]. For Internet companies, it is necessary to learn more about the interests and hobbies of users [16]. Users are unable to analyze and choose from numerous tourism products; therefore, a suitable recommendation system is urgently needed that can solve this problem. Such a recommendation system will build a user model based on the data and identify the user’s interests and hobbies. Then, by comparing recommended items, the system can provide users with accurate product information [17]. The most used technology is collaborative filtering, which can be applied on various occasions and can achieve excellent results. Fig 1 shows that the system is divided into three parts: user, object, and algorithm [18]. The first part identifies the user’s interests and hobbies from information such as consumption data, search data, and browse data. The algorithm and object identify and compare products provided by merchants, match the hobbies of users on the e-commerce platforms, and recommend products with the highest scores to users.

**Fig 1:** The structure of a tourism collaborative recommendation system.

Moreover, if a user provides little data, it will be difficult for this user to get recommendations. After all, the number of people traveling is a minority. Therefore, in tourism service recommendations, the problem of data sparsity is very prominent, and it is difficult to achieve excellent results using traditional collaborative filtering technology [19].

(2) Internet information technology: the operation mode of the tourism service supply chain, with travel agencies as the core, has occupied the mainstream of the tourism consumption market for a long time. However, this mode has gradually exposed some shortcomings in the long-term operation process. For example, tourism enterprises heavily on package tour contractors, but the coordination between them is insufficient; tourism service products are single, and tourists can only passively accept the existing tourism products provided by travel agencies, which affects and hinders the personalized development of tourist demand and the reform and innovation of the tourism industry. More tourism enterprises encapsulate their business into Web services and publish them on the Internet based on the advancement of Internet information technology and the rapid popularization of the Internet. As individual travel and self-guided travel continue to heat up, people have become accustomed to using these online services for travel planning and services purchasing. Some travel e-commerce websites have stood out in the fierce competition in the tourism industry, which has become recognized by the industry and known to most tourists as famous brands. However, the academic circle of supply chain management has not yet been able to put forward complete theoretical support for this new type of tourism business model, and whether this model can be improved has not received enough attention so far.

### 2.2 Principle of the deep recommendation model

(1) Principle of CNN: This is a feedforward neural network. It is a deep learning algorithm that can quickly respond to and process information by establishing a network system based on the principle of human neurons [20]. It consists of convolution layers and information collection layers alternately to form a network topology [21]. CNN uses the method of backpropagation to realize the transmission of information. The specific calculation of the feature extraction process is shown below. The cross-entropy loss function for the classification error of the *i* sample (*x*_*i*_,y_i_) (is defined as follows.

$$L_{i}=-\ln e^{{\text{s}}_{y_{i}}}+\ln\sum e^{s_{i}}$$ (1)

The output of the sample (*x*_*i*_,y_i_) after the convolution layers is *f*(*x*). Then, the corresponding loss value should be as follows.

$$L_{i}(f(x),y)=-\ln f{\left(x\right)}_{y}$$ (2)

The error-sensitive items of the output layer of the CNN deep learning *l* layer are as follows.

$$\delta_{l}=\frac{\partial L}{\partial a^{l}}=\nabla_{a}^{l}(x)-\ln f{\left(x\right)}_{y}=f(x)-y$$ (3)

Where $S_{x_{i}},S_{{\text{y}}_{i}}$ is the score function, ∂*L* is the derivative of the convolution nerve of the *l* layer, *a*^*l*^ represents the input of the layer *l*. The convolution layer uses its convolution kernel to convolve with the input image and output its feature map through the neuron activation function, thereby realizing the feature extraction of the input image. The convolution process is defined as follows.

$$x_{j}^{l}=f(\sum_{i\in M_{j}}x_{i}^{l-1}\times k_{ij}^{l}+b_{j}^{l})$$ (4)

Where *l* is the number of convolution layers in the model, $k_{ij}^{l}$ represents the number of convolution kernels, $b_{j}^{l}$ represents the additive bias, *f* represents the activation function, and *M*_*j*_ represents the input image. The specific structure is shown in Fig 2.

**Fig 2:** Process of deep learning CNN.

(2) CNN application: Fig 3 shows the network structure of the review information of users and scenic spots. In this structure, the user review information network has a network architecture based on CNN, which is adopted because CNN has a good effect on the hidden feature extraction of text information. For the review information of tourism service items, its vector-matrix is obtained, which is used as network input. This network is equivalent to the parallel structure of the user review information network. Finally, through this network, the features of the review information of tourism service items are obtained. Other information is passed through an algorithm similar to DNN. In addition to the input layer and the output layer, the multi-layer perceptron includes at least one hidden layer, which is similar to a neural network model with multiple hidden layers.

**Fig 3:** Network structure of the review information of users and scenic spots.

(3) Principle of DNN: this is a neural network with multiple hidden layers based on the extension of the perceptron [22]. DNN is divided according to the position of different layers. The neural network layers inside the DNN can be divided into three categories: the input layer, the hidden layer, and the output layer, as shown in the figure below. Generally, the first layer is the input layer, the last layer is the output layer, and the middle layers are all hidden layers [23]. The specific structure is shown in Fig 4. For DNN, the most important thing is the perception of the input value. The specific perception calculation is as follows.

$$Output=\left\{ \begin{array}{l} 0\;if\sum {}_{j}\omega_{j}x_{j}\leq thread\\ 1\;if\sum {}_{j}\omega_{j}x_{j}>thread \end{array}\right.$$ (5)

Where Σ_j_*ω*_*j*_*x*_*j*_ is the integration of the assigned weights, and the *thread* is a real number of perception thresholds. Another feature of CNN is that the included neurons are S-type neurons, which can transmit information in multiple directions. The function *δ*(*z*) is defined as follows.

$$\delta (z)=\frac{1}{1+e^{-z}}$$ (6)

**Fig 4:** Structure of DNN.

(4) DNN application: the construction of the neural network is based on TensorFlow. Fig 5 shows that the model is divided into three parts: review information network of tourists; review information network of tourism service items; and other information networks. The data input to the model is all sorted and cleaned. These data are also divided into three parts. After these data pass through the neural network model, the feature parts will be extracted and described abstractly. A synergy layer is added on top to enable the features extracted by the three parts to influence each other. The features extracted from the three parts are integrated to make the final score prediction.

**Fig 5:** Deep prediction model framework.

### 2.3 Tourism recommendation algorithm

A comparative investigation is conducted with other tourism service models to verify the effectiveness of the proposed method. It mainly uses three algorithm models: Matrix Factorization (MF), Probabilistic Matrix Factorization (PMF), and Latent Dirichlet Allocation (LDA).

(1) The first method is the recommendation method of the traditional latent factor model, i.e., MF. It is an algorithm based on low-rank matrix factorization. Koren proposed this method in 2008, and it has become the most widely used collaborative filtering method. It only uses the scoring matrix as input to estimate two low-rank matrices and perform score prediction. For a given user, the scoring of the item can be expressed as follows.

$$\eta_{\text{ui}}\text{=}\mu {\text{+b}}_{\text{i}}+b_{u}+q_{i}p_{u}$$ (7)

Where *μ* represents the average scoring value of the item, b_i_ represents the offset of the item, *b*_*u*_ represents the offset of the user, and *q*_*i*_*p*_*u*_ represents the interaction between the user and the item; that is, the user’s overall interest in the item. Then, the minimum objective function is as follows.

$$E={\sum_{b*,q*,p*(u,i)\in \kappa }\left(\gamma_{ui}-\eta_{ui}\right)}^{2}+\lambda (b_{i}{}^{2}+b_{u}{}^{2}+{\left\|q_{i}\right\|}^{2}+{\left\|p_{u}\right\|}^{2})$$ (8)

In (8), *γ*_*ui*_ represents the actual scoring result of the item, *q*_*i*_ represents the user’s interaction value, *q*_*i*_ is the item’s interaction value, and b*,q*,p*(*u*,*i*) represents the offset of the item and the user under the value of *i*.

(2) The second method is the PMF, which is essentially matrix factorization. However, it uses Gaussian distribution to model the hidden factors of users and items. Traditional matrix factorization, such as SVD, starts from the perspective of optimization goals. The PMF explains the hidden factors between users and items from the perspective of probability generation. The idea of PMF is based on the linear factor model, which uses the coefficients related to the user to model the user’s hobbies as a linear combination of a series of vectors. If the score is a normal distribution that conforms to Gaussian noise, it has the following equation.

$$p(R|U,V,\delta^{2})=\prod_{i=1}^{N}\prod_{j=1}^{M}{\left[\sigma (R_{ij}|U_{i}^{T}V_{j},\sigma^{2})\right]}^{I_{ij}}$$ (9)

Where $\sigma (R_{ij}|U_{i}^{T}V_{j},\sigma^{2})$ represents the probability density function of the Gaussian distribution,*I*_ij_ represents the indicator function. If the user *i* scores the item *j*, the result is either 1 or 0. The Gaussian of the hidden vector of each user and item with an average value of 0 is verified, then:

$$p(R|\delta_{U}{}^{2})=\prod_{i=1}^{N}\sigma (U_{i}|0,\sigma_{U}{}^{2}I)$$ (10)

$$p(R|\delta_{V}{}^{2})=\prod_{i=1}^{N}\sigma (U_{\text{j}}|0,\sigma_{V}{}^{2}I)$$ (11)

Then, according to Bayes’ rule, the post-test probability of the hidden factors U and V can be obtained as follows.

$$p(U,V|R,\delta_{U}{}^{2}\delta_{V}{}^{2}\delta^{2})\propto p(R|U,V,\delta^{2})p(U|\delta_{U}{}^{2})P(V|\delta_{V}{}^{2})$$ (12)

After removing the logarithm, the minimum objective function is as follows.

$$E\text{=}\frac{1}{2}\sum_{\text{i=1}}^{N}\sum_{j=1}^{M}I_{i,j}(R_{i,j}-U_{i}^{T}V_{j})2+\frac{\lambda_{U}}{2}{\sum_{i=1}^{N}\left\|U_{i}\right\|}_{F}^{2}+\frac{\lambda_{V}}{2}{\sum_{j=1}^{M}\left\|U_{j}\right\|}_{F}^{2}$$ (13)

(3) The third method uses the document topic generation model for the recommendation. LDA is a famous topic model generation algorithm. LDA associates documents with K-dimensional topic distribution and encodes the discussion of K topics in some words in the documents; that is, how likely it is that the words in the document discuss the topic. The model can be defined as follows.

$$p(\nu |\theta ,\phi ,z)={\prod_{d\in \nu }\prod_{j=1}^{N_{d}}\theta_{zd,j}\phi }_{zd,j,\omega dj}$$ (14)

In the experiment, LDA is used to learn the topic distribution from a set of reviews for each item. The distribution of topics learned is considered to describe the potential features of each item. Then, the gradient descent is used to optimize the score prediction accuracy to estimate the potential features of each user. The objective function is as follows.

$$f(\nu |\theta ,\alpha ,\kappa ,z)={\sum_{\gamma_{u,i}\in \nu }\left(rec(u,i)-\gamma_{u,i}\right)}^{2}-\mu l(\nu |\theta ,\alpha ,z)$$ (15)

Where *V* represents the learning topic, *θ* represents feature 1, *α* represents feature 2, *K* represents feature 3, *z* represents feature 4, *rec*(*u*,*i*) represents the accuracy of scoring prediction, *γ*_*u*,*i*_ represents user scores, and *μl*(*ν*|*θ*,*α*,*z*) represents the descent gradient value.

(4) Factorization machine: It is the best processing algorithm to solve data sparsity, usually with a non-linear kernel function. It is specifically designed independently for different problems. Also, it can model and evaluate the interaction between different types of variables, thereby improving the prediction accuracy of the model.

Since MF has only a single matrix, there will be a significant error in the prediction of the score. PMF models the user’s hobbies as a linear combination of a series of vectors by adding Gaussian distribution. In this way, subsequent data processing needs to convert vectors into data before modeling, which will occupy much system memory, and the operation efficiency of the algorithm will be reduced. LDA, which uses the document topic generation model for the recommendation, builds a model with the aid of K-dimensional topic distribution. Although the algorithm is efficient, the accuracy of the system is low, and the problem of data sparsity still exists. After analysis, it is found that these traditional algorithms cannot effectively solve the problem of data sparsity. Therefore, the tourism recommendation system based on the Internet and deep learning technology is proposed. The system innovatively integrates Convolutional Neural Network (CNN) and Deep Neural Network (DNN) algorithms, adds word embedding technology to data processing, and adds factorization technology to deep learning. Through the integration of multiple technologies, the interaction between users and tourism service items is deeply explored. It effectively solves the problem of data sparsity, thereby improving the performance of the tourism recommendation service system.

Some variants of the deep model are proposed to prove the effectiveness and advantages of such a combination.

User model: the review network that processes tourism service items in CDMF (CNN-DNN Embedding Factorization) is replaced with a matrix, which is randomly generated.

Reviews model: this model only retains two CNNs that process text information of user reviews and tourism service reviews. It does not use a DNN that processes necessary information about users and tourism service items. It is equivalent to just using the review text information of users and tourism service items to make recommendations.

DNN model: this is a DNN that only retains and processes various necessary information of users and tourism service items. It does not use CNN that processes review text information of users and tourism service items.

Item model: the network that processes user review information in CDMF is replaced with a matrix. This matrix is also randomly generated; that is, this model cannot use user review text information.

TFIDF: this uses the TFIDF algorithm instead of the word embedding method to characterize text information.

### 2.4 Construction of deep learning recommendation system

Aiming at the data sparsity of the original tourism recommendation system and the drawbacks of traditional algorithms, a tourism service recommendation model based on deep learning is proposed. Neural network technology is used to build a deep prediction model. This model uses the review information of users and tourism service items as well as their necessary information to learn the hidden features shared by users and tourism service items. It can deeply mine the interaction between users and tourism service items, effectively solving the problem of data sparsity, and thereby improving the performance of recommendation.

The proposed model implementation framework is divided into four main modules: data collection and processing, deep recommendation model construction (CNN-DNN), network training, and recommendation list generation. The overall design of the concrete model is shown in Fig 2. This model builds an interaction network between users and tourism service items by using the relationship between them on the Internet (review information and corporate evaluation). By means of the factorization and embedding methods, the recognition and classification of information are improved, thereby effectively improving recommendation performance. It is named CNN-DNN Embedding Factorization (CDMF).

The process of the proposed model is shown in Fig 6, which is divided into four steps: (1) data collection, including consumption data, travel data, search data, and browsing data; (2) data preprocessing by word embedding technology; (3) model construction; specifically, these processed data are entered into the data end of the neural network to build a neural network model through factorization; (4) recommendation; through the training of the neural network, the tourism service is effectively recommended to a user according to this user’s interest and hobby. The entire process is referred to as CDMF.

**Fig 6:** Overall framework of tourism service recommendation model based on Internet information technology and deep learning.

### 2.5 Data collection and processing

(1) Data collection: In this experiment, data are collected using the distributed web crawler framework implemented by Scrapy+redis+MongoDB, which uses Internet information technology to collected network data and convert the collected data into Json format, the number of users in the dataset was 206,387, the number of scenic spots was 7,300, and the number of reviews was 1,283,715. The users’ information includes gender, age, occupation, city, historical review items, and review data. The behavior features of the user are extracted to analyze user hobbies and build the feature model. The tourism service information includes the name, location, label, and review data of the tourism service items. The attribute features of the tourism service item are extracted to construct the feature model of the tourism service item.

(2) Data processing: word embedding technology was used to process data. This refers to embedding a high-dimensional space whose dimension is the number of all words into a continuous vector space with much lower dimensions. Each word or phrase was mapped to a vector on the real field [24]. The specific structure is shown in Fig 7. Chinese word segmentation technology was used for processing the review text information of users and items. At the same time, this technology can calculate sufficient distance between two words, as well as describing the semantic distinctions between words. It is an effective method for processing text information. Here, this method is mainly responsible for filtering spam reviews, mood reviews, and some unimportant special symbols.

**Fig 7:** Model structure of word embedding technology.

### 2.6 Model training and indicator detection

The following indicators are used for analysis to determine the stability of the system score. In the investigation of recommendation systems, prediction accuracy is a frequently discussed attribute. The recommendation system generally uses a prediction engine to predict the user’s score or probability of using items. Here, the proposed method generates a prediction score for the user-tourism service item and a personalized recommendation list according to the ranking of the score. Therefore, these two results are evaluated to verify the performance of the method. The Mean Squared Error (MSE), Mean Absolute Deviation (MAE), and Pre (Precision), which are often used to evaluate the prediction accuracy of the recommendation system, are adopted to evaluate the accuracy of the prediction score. Mean Average Precision (MAP) is used to evaluate the accuracy and sensitivity of the generated recommendation list. The specific equation is as follows. The dataset is divided into three groups: training set, validation set, and test set. For each dataset, 80% is used as the training set, 10% as the validation set for hyperparameter adjustment, and 10% as the test set.

(1) MSE is the mean value of the sum of squared errors of the corresponding points between the predicted data and the original data. The specific equation is as follows.

$$MSE=\frac{1}{N}{\sum_{n=1}^{N}\left(\gamma_{u}{}_{i}-\eta_{ui}\right)}^{2}$$ (16)

(2) MAE is a measure of the error between paired observations of the same phenomenon. The specific equation is as follows.

$$MAE=\frac{1}{N}\sum_{n=1}^{N}\left|\gamma_{u}{}_{i}-\eta_{ui}\right|$$ (17)

Where *u* is the user for centralized testing, *i* is the tourism service item, *η*_*ui*_ represents the prediction score generated by the recommendation algorithm, *γ*_*ui*_ represents the actual scoring of item *i* by the user *u*, and N is the number of observations in the test set. When the accuracy of the algorithm is higher, the values of *η*_*ui*_ and *γ*_*ui*_ are closer. Then, the values of MSE and MAE are lower.

(3) Pre is the true, correct proportion in all predictions. Personalized recommendations for each user are sorted and generated according to the predicted scores. Therefore, the accuracy needs to be used to measure the quality of the generated list. The specific equation is as follows.

$$\text{Pr}ecision=\frac{\sum {}_{u\in U}\left|R(u)\cap T(U)\right|}{\sum {}_{u\in U}\left|R(u)\right|}$$ (18)

Where *R*(*u*)is the recommended list for the user, *T*(*U*) is the list of reviews made by the user.

(4) MAP is obtained by comprehensively weighting the average precision (AP) of all categories detected. The specific equation is as follows.

$$AP\text{=}\frac{\sum {}_{\text{k=}1}^{N}P\text{@k}\times I}{\left|R\right|}$$ (19)

Where *N* represents the length of the recommendation list, |*R*|is the number of items of behavior that the user generates in the test set, *P*@k represents the precision of the recommendation list at k, and *I* represents whether the item at this position is an item that is generated as user behavior.

## 3. Results and discussion

### 3.1 Performance comparison of different models

Both ANN and CNN have smaller MAE and MSE values, whether it is in the training set or the test set compared with the separate network models, as shown in Fig 8. The proposed CDMF has the lowest error in the prediction score, representing the high accuracy of the model. Although the effect of PMF is better than that of MF, compared with the proposed CDMF, neither of these two methods achieves the desired performance. This is mainly because neither of these two methods can use other information except scoring information, such as review text information, disabling them to mine more information from the review text. Hence, considering review text information can improve the accuracy of score prediction. LDA utilizes review text information for learning some features from reviews to improve the prediction accuracy. However, Fig 8 suggests a big gap compared with the proposed CDMF. This is because LDA’s modeling process of review texts is independent of scoring, making it challenging to ensure that the learned features are conducive to score prediction. Based on the above results, the proposed tourism service recommendation model combining Internet information technology with deep learning has high accuracy.

**Fig 8:** Performance analysis of MAE and MSE of different models.

Fig 9 shows that the CDMF method can maintain excellent precision when generating a personalized recommendation list for users. The sensitivity and accuracy of the recommendation list are better than other algorithms. The proposed CDMF method can still maintain good performance when generating a personalized recommendation list for users, and the sensitivity and accuracy of the recommendation list remain the first among the four algorithms. Compared with other algorithms, CDMF can make fair use of some primary information and review text information, as well as the hidden interaction relationship between this information, which is not available in other algorithms. Therefore, the accuracy and sensitivity of the generated recommendation list are lower than the DPMR algorithm. Therefore, the above results illustrate the feasibility of the proposed system for tourism service recommendations.

**Fig 9:** Performance analysis of pre and MAP of different models.

### 3.2 Improved model performance analysis

Fig 10 shows that, when CNN and ANN are not used, the model recommendation efficiency is significantly different. In the training set, using the DNN can improve the precision of the model by 30%, and using the embedding method can improve the accuracy by 33.3%. Using the factorization machine can significantly improve the precision of the algorithm, with an improvement effect of 40%. The Item and User model is a variant of the User model, which replaces the network that processes reviews on travel service items in the CDMF with a randomly generated matrix. The Item and User model is also a variant of the Item model variant, which replaces the network that processes user review information in the CDMF with a matrix. This matrix is also randomly generated. The Item and User model only considers the review text of the user and one of the travel service items, and cannot learn from the user. The interaction with the review text of travel service items is consistent with the results of the training set on the test set. The Reviews model can obtain better results than Item and User, but it still cannot reach the performance of CDMF. This is because the Reviews model’s modeling of the interaction between users and travel service items only considers the review text information of users and travel service items rather than other primary information of users and travel service items as CDMF does. The results of CDMF-DNN are not as good as those of CDMF, which also shows that only considering the primary information of users and travel services and ignoring their review text information cannot obtain good results. Therefore, the proposed DNN-CNN parallel network analysis and the CDMF model combining the embedding method with the factorization machine consider the review text information of users and tourism service items. Also, they have a significant effect on improving the precision of recommendations.

**Fig 10:** Impact of the improved model on prediction results.

### 3.3 Determination of optimal model parameters

Practical experience suggests that three significant parameters affect the model. One is the number of hidden factors in the factorization machine, the second is the number of convolution kernels in CNN, and the third is the size and the number of neurons in the neural network. Fig 11 illustrates that, as the number of hidden factors increases, the precision of the model continues to improve. When the number of hidden factors reaches 40, the precision of the model reaches the lowest value. As the number of convolutions increases, the precision of the model continues to improve. When the number of convolution kernels reaches 100, the MSE of the model reaches the lowest; above 100, the performance of the model no longer improves. Increasing the depth and width of the hidden layer can improve the effect, but after a certain point, the effect will not increase significantly, and the amount of calculation will become increasingly larger. Increasing the depth and width of the hidden layer can improve the effect; however, the effect will not increase significantly, and the amount of calculation will become larger. Therefore, after comprehensive consideration, the two-layer combination of 100 ReLU + 50 ReLU is selected as the configuration of the DNN network. After measuring under this parameter, the model has the highest precision.

**Fig 11:** Impact of different model parameters on prediction results. A1 is 25 hidden layers, A2 is 50 hidden layers, A3 is 100 hidden layers, A4 is 50 first hidden layers + 25 second hidden layers, A5 is 100 first hidden layers + 50 second hidden layers, A6 is 100 first hidden layers + 50 second hidden layers + 25 third hidden layers.

## 4. Conclusion

According to the traditional collaborative filtering algorithm, a deep-learning-based recommendation model for tourism services under Internet information technology is proposed. This method uses neural networks to mine potential hidden features among users and tourism service items. Three parallel networks are constructed through word embedding and factorization machine technology. The user and item review text information, as well as other information, are separately processed, which alleviates the sparsity of user information and effectively improves the accuracy of the model. The user’s scores of tourism service items are predicted through the network. Next, the predicted scores are sorted to generate a recommendation list for personalized recommendations. Although some progress has been made, several shortcomings need to be improved: (1) Product recommendations for tourism services are affected by seasons. The amount of products that people need during the peak travel season increases sharply, but there are few product outputs during the off-peak season, which is not considered in the modeling. In the off-peak season, the model is established solely through user reviews. (2) In the process of recommending travel products, the most crucial thing is word of mouth. Therefore, it is essential to understand the social relations of users effectively. This is one of the critical factors affecting tourism travel but is also not considered in the modeling. (3) When collecting tourism product data, not only textual information but also many images are collected. Currently, more users value images because images are more realistic; however, the processing of images is not analyzed. In the future, an in-depth investigation of these areas will be conducted to enrich the user’s feature information and improve the accuracy of recommendations.

## Supporting information

S1 Data (ZIP)
